# Ethnomedicinal Use, Phytochemistry, and Pharmacology of *Xylocarpus granatum* J. Koenig

**DOI:** 10.1155/2021/8922196

**Published:** 2021-08-30

**Authors:** Dipta Dey, Cristina Quispe, Rajib Hossain, Divya Jain, Rasel Ahmed Khan, Pracheta Janmeda, Muhammad Torequl Islam, Hafiz Ansar Rasul Suleria, Miquel Martorell, Sevgi Durna Daştan, Manoj Kumar, Yasaman Taheri, Anka Trajkovska Petkoska, Javad Sharifi-Rad

**Affiliations:** ^1^Department of Biochemistry and Molecular Biology, Life Science Faculty, Bangabandhu Sheikh Mujibur Rahman Science and Technology University, Gopalganj 8100, Bangladesh; ^2^Facultad de Ciencias de la Salud, Universidad Arturo Prat, Avda. Arturo Prat 2120, Iquique 1110939, Chile; ^3^Department of Pharmacy, Life Science Faculty, Bangabandhu Sheikh Mujibur Rahman Science and Technology University, Gopalganj 8100, Bangladesh; ^4^Department of Bioscience and Biotechnology, Banasthali Vidyapith, Vanasthali, India; ^5^Pharmacy Discipline, Khulna University, Khulna, Bangladesh; ^6^Department of Agriculture and Food Systems, The University of Melbourne, Melbourne 3010, Australia; ^7^Department of Nutrition and Dietetics, Faculty of Pharmacy, and Centre for Healthy Living, University of Concepción, Concepción 4070386, Chile; ^8^Universidad de Concepción, Unidad de Desarrollo Tecnológico, UDT, Concepción 4070386, Chile; ^9^Department of Biology, Faculty of Science, Sivas Cumhuriyet University, Sivas 58140, Turkey; ^10^Beekeeping Development Application and Research Center, Sivas Cumhuriyet University, Sivas 58140, Turkey; ^11^Chemical and Biochemical Processing Division, ICAR–Central Institute for Research on Cotton Technology, Mumbai 400019, India; ^12^Phytochemistry Research Center, Shahid Beheshti University of Medical Sciences, Tehran, Iran; ^13^Faculty of Technology and Technical Sciences, St. Kliment Ohridski University, Bitola 1400, North Macedonia

## Abstract

The mangrove plants are the potential sources of foods and remedies for people living in the forests and nearby communities. *Xylocarpus granatum* J. Koenig is traditionally used to treat various diseases including diarrhea, cholera, dysentery, fever, malaria, and viral infections, among others. To summarize critically the taxonomy, ethnomedicinal, phytochemistry, and pharmacological activities of *X. granatum*, information was collected from different databases. An up-to-date search (till June 2020) was carried out with the help of various scientific web resources from databases such as PubMed, Science Direct, Google Scholar, and various patent offices (e.g., WIPO, CIPO, and USPTO) using the keywords “*Xylocarpus granatum*” and then paired with ethnomedicinal use and phytochemical, phytochemistry, and pharmacological activity (*in vitro, ex vivo*, and *in vivo* studies). Findings revealed that seeds, fruits, stem bark, leaf, and twigs of *X. granatum* exhibited a wide range of key phytochemicals including limonoids, phragmalin, limonoid-based alkaloids, mexicanolides, protolimonoids, flavonols, and lactones. The plant possessed potent antioxidant, anticancer, antidiabetic, antimicrobial, antimalarial, antifeedant, and neuroprotective activities. No clinical studies have been reported in the databases. Ethnomedicinal assessment indicated the application of *X. granatum* in various fields of medical science specially to treat various human ailments, and this was attributed to the presence of enormous alkaloids as confirmed by pharmacological studies. However, to understand the mechanism of action in-depth studies are required. In view of these findings, more research is necessary to explore and characterize the chemical compounds and toxicological aspects of this medicinal mangrove plant. Overall, it can be stated that *X. granatum* may be one of the hopeful medicinal herbs for the treatment of various diseases in human beings.

## 1. Introduction

Traditional medicines like Chinese traditional medicine, Ayurveda, Unani, and Korean traditional medicine have been used extensively ever since the ancient times. These medicines are based on using natural products for treating various human ailments [1]. Use of new medicines with no doubt helps treat different diseases, but it also poses a risk of side effects. Increased demands for reducing these side effects of the current drugs are driving researchers and pharmacologist towards formulating natural plant-based drugs, thereby exploring different traditionally used medicinal plants/herbs [1]. *Xylocarpus granatum* J. Koenig is a good example of a medicative plant that is used as a traditional herbal drug [2]. *X. granatum* is a species of the mahogany family and is widely distributed in the coastal forests of Bengal, Burma, Malay Peninsula, Andaman, and Africa. In Bangladesh, this plant is found in low lying, a swampy locality in the Sundarbans mangrove forest [3]. It is spread across the coastal areas of tropical and subtropical zones and river delta. Typically, this plant's different parts are used for different purposes, most popularly used for the treatment of diarrhea, dyslipidemia, fever, inflammation, malaria, cholera, dysentery, and so on [4, 5]. Various types of chemical compounds are extracted from the different parts of the plant such as limonoids, phragmalin, limonoids based alkaloids, mexicanolides, protolimonoids, flavonol-like compound, lactone, ethanol extract, methanol extract, and alkaloids, among others [6, 7]. Limonoids are the most vital chemical component that is isolated from the different parts of the *X. granatum* plant [8]. Numerous limonoids are isolated from different parts of *X. granatum* such as fruit peel, seed kernels, seed, fruit, and seed coat [9]. Limonoids possess diverse pharmacological activities, such as antimicrobial, antimalarial, antiviral, anticancer, antidiabetic, antioxidant, antifeedant [10], and neuroprotective effects [11]. Other potential activities *X. granatum* extracts include antifilarial, antidepressant, antimalarial [12], and antisecretory effects [13]. So, the limonoids are important pharmacologically active constituents of *X. granatum* fruit that need to be exploited further [9]. A more detailed investigation need to be done on the toxicological effects and clinical trials on humans.

This review offers up-to-date information on the phytochemical profile and biopharmacological effects of *X. granatum* on the basis of scientific reports found in the databases.

## 2. Research Methodology

The literature on *X. granatum* botanical description, ethnomedicinal uses, secondary metabolites, and biological properties was collected, analyzed, and summarized in this review. Scientific search engines, such as PubMed, ScienceDirect, SpringerLink, Web of Science, Scopus, Wiley Online, SciFinder, and Google Scholar, and various patent offices (e.g., WIPO, CIPO, and USPTO), were used to collect all published articles about this species. Several terms were used as keywords like *Xylocarpus granatum*, chemical compounds and *Xylocarpus granatum*, taxonomical classification, antidiabetic and *Xylocarpus granatum*, and limonoids and their pharmacological activity. All published work on *X. granatum* in different languages (English) was cited in this study. The identification and examination of the collected manuscripts were based on their titles and abstracts. Reference lists of the retrieved papers were also examined to identify further relevant papers. Chemical structures were drawn using ChemSketch version 12.01 software.

## 3. Result and Discussion

### 3.1. Botanical Description

The word *Xylocarpus* means woody fruit (in Latin) and refers to the large and distinctly woody fruit and seeds of this genus. *X. granatum* taxonomical classification is given as follows [14]. The maximum height of the *X. granatum* is 12 m (39 ft); it is a small to medium-sized evergreen tree. The evergreen leaves of the tree have special characteristics; the leaves are pinnate and arranged spirally on the twigs (Figure 1). The trunk has buttresses and above-ground roots, which extend for long distances to either side. *X. granatum* flowers are white or pinkish-yellow; each flower is 8 mm wide with four parts. The flowers are produced spherical, large, woody capsules, 9–12 cm in diameter. If the capsules are split, this brings out a dozen seeds.

### 3.2. Taxonomy and Geographic Distribution

The taxonomical classification of *X. granatum* [14] is as follows:

  Kingdom: Plantae
  Phylum: Magnoliophyta
  Class: Eudicots
  Order: Sapindales
  Family: Meliaceae
  Genus: *Xylocarpus*
  Species: *Xylocarpus* g*ranatum* J. Koenig

*X. granatum,* a species of mangrove in the mahogany family (Meliaceae), is commonly known as “cannonball mangrove, cedar mangrove [15], dhundul [16], or puzzle nut tree” [17]. Asia, Africa, Australia [18], and the Pacific Islands are the main inhabitant of this plant [15]. This plant is found in low lying, swampy locality in the Sundarbans mangrove forests in Bangladesh [3]. This forest covers 6017 km^2^ in Bangladesh and mangroves are salt-tolerant forest ecosystems of tropical and subtropical intertidal regions of the world [3]. This plant extends from Tanzania, Kenya, and Mozambique to Malaysia, Indonesia, Thailand, Papua New Guinea, India, Bangladesh, and northern Australia [3]. This species is native to the tropical and subtropical western Indo-Pacific region [19].

### 3.3. Ethnopharmacological Uses

*X. granatum*, a puzzle nut tree, is a mangrove species belonging to mahogany family [20, 21]. It is commonly known as “pussur” in Hindi and “dhundul” in Bengali. It is an evergreen tree having moderate-sized grey bark, usually growing in coastal forests of Bengal, Burma, the Malaya peninsula, Andaman Islands, and island of Australia and Africa [12]. It is a medicinal plant and used by different ethnic communities all over the world [22]. Several reports suggested that from past to present this plant has significant medicinal properties [23]. *X. granatum* plants have several bioactive compounds, including gedunin and limonoids [6, 24]. All of these compounds possess significant inhibitory activity against cancer [16, 25] and malarial, viral, feedant, diabetes, filarial activity, and fungicidal activity from ancient times [10, 26]. All of these compounds extracted from the twigs and leaves, fruits, seeds, barks, seed kernels, and stem bark.

In the previous studies, researchers present various traditional uses of *X. granatum* extract. In southeast Asia, it is used as a treatment of diarrhea, fevers such as malaria, viral diseases like influenza, and cholera and also as an antifeedant or insecticide throughout ancient times [8, 25]. In folklore, the *X. granatum* plant has been applied to treat malaria, fever, cholera, dysentery, and diarrhea in many countries including India. The extraction of leaves, fruits, and barks of *X. granatum* possesses potential free radical scavenging activities [4]. Besides, Uddin et al. [16] proposed that this plant extract chemicals have a variety of medicinal properties and in Bangladesh, and it was employed for the treatment of fever, malaria, cholera, diarrhea, and dysentery. Also, antioxidant and antifilarial activities have been reported from ancient times [16].

### 3.4. Phytochemistry

The *X. granatum* plant contains several bioactive constituents (Table 1 and Figure 2). Limonoids are the most vital chemical component that are isolated from the different parts of the *X. granatum* plant [8]. Moreover, *X. granatum's* seeds consist of sundarbanxylogranins A–E [27]; krishnagranatins A–I [28]; thaixylogranins A–H [29]; granaxylocarpins A–E [30]; xylocarpanoids A and B [31]; xylomexicanins A–D, I, and J [32–34]; xyloccensins I, K, L, O–S, V, W, and Y [10, 12, 35, 36]; hainangranatumins A–J [37]; xylogranatins F–R [38]; thaigranatins A–E [39]; xylocartin C [40]; andhraxylocarpins A–E [41]; protoxylogranatin A-B [42, 43]; protoxylocarpins F–H [25].

The plant fruit contains gedunin [16, 40], andirobin, mexicanolide, and phragmalin [40]; cipadesin A [2]; xylocarpins A-I [8]; photogedunin [48]; xylocarpin L [35]; xyloccensin I, Y, X1, X2 [49]; xylogranatin E [50]; xylogranatinin [51]. Furthermore, stem bark of *X. granatum* consists of xyloccensin M and N [44]; xyloccensins Q–U [10]; xyloccensin L [45]; xyloccensin I and J [46]; xyloccensins O and P [47]. Leaf and twigs contain lactone [22]; xyloccensins O–S and V [36]; xylogranin B [26]; xylogranatopyridines A and B [52]; xylogranatumines A–G [53]; xylogranatin E [50], and root bark contains N-methylflindersine [54].

It is evident that *X. granatum* is rich in various compounds, but limonoids, which is an oxidized tetranortriterpenoid derivative, is most dominant and widely studied secondary metabolite. This group of compounds is gaining more and more interest of scientific community due to its various health promoting effects. There are as many as 100 limonoids that are extracted and characterized. Limonoids have important biological activities such as anticancer, antioxidant, antiulcer, antimicrobial, and antiviral actions [55]. Traditionally, these mangroves are also used to treat the troubles caused by dysentery, diarrhea, and abdominal pains [48]. In a recent study, 25 new limonoids have been detected using high resolution electrospray ionization mass spectroscopy (HRESIMS) in *X. granatum* of Hainan mangrove region. The structures of these compounds were also established using single-crystal X-ray diffraction analyses, nuclear magnetic resonance spectroscopy, and electronic circular dichroism spectra. Limonoids showed typical bridges of C_3_-O-C_8_ and C_1_-O-C_8_ in mexicanolides, whereas few compounds, which are derivatives of azadirone, showed C_1_-O-C_29_ bridges (Zahang et al., 2020).

### 3.5. Pharmacological Investigation

The pharmacological activities of *Xylocarpus granatum* J. Koenig are summarized in Table 2.

#### 3.5.1. Anticancer Activity

Cancer is the abnormal proliferation of the human body's cells. The uncontrolled development of normal cells can initiate cancer. In recent studies, the anticancer properties have been found in some plant extracts and their isolated compounds developed by the researchers. Amongst them is *X. granatum*, a well-known mangrove plant, a rich source of bioactive compounds, such as protolimonoids (apotirucallanes) [57, 58], gedunin [16], xylogranatumines A–G [53], protoxylocarpins F–H [25], and so on, which showed anticancer activity. Besides, protolimonoids exhibited a wide range of bioactivities, including insecticidal [59], and CDC25B (M-phase inducer phosphatase 2) inhibitory properties [60]. The cytotoxic activity of gedunin extracted from bark of *X. granatum* demonstrated moderate levels of anticancer activity in colon cancer cell lines with IC_50_ value of 16.83 µM concentration. In this study, gedunin moderately inhibited CaCo2 (human colorectal adenocarcinoma) and had growth inhibitory activity [16]. Moreover, xylogranatumines A–G (apotirucallane protolimonoids) had the potential to cytotoxic activities against human A549 (lung adenocarcinoma) tumor cell line. However, at 10 *μ*M concentration, only xylogranatumine F showed weak cytotoxic activity against A549 alveolar tumor cell with inhibition of 54.2% at the concentration of 10 *μ*M, while others were inactive (<50% inhibition at 10 *μ*M) [53]. Besides, the isolated protoxylocarpins F-H from seed kernels were assessed for cytotoxicity activity against five human tumor cell lines. However, only 7-deacetylgenudin showed cytotoxic activity against lung cancer cell line, that is, CHAGO (IC_50_: 16.0 *µ*M), and hepatocarcinoma cell line, Hep-G2 (IC_50_: 10.26 *µ*M), while xylogranatin C showed cytotoxic activity against CHAGO cells (IC_50_: 9.16 *µ*M) and 7-oxo-7-deacetoxygenudin depicted anticancer activity against Hep-G2 cells (IC_50_: 16.17 *µ*M) [25]. In human breast carcinoma cells (KT), xylomexicanin A extracted from seed exhibited antiproliferative at IC_50_ value of 7.43 *µ*M [32], and xylomexicanin F showed moderate antiproliferative activity against human tumor cell lines A549 and RERF at 18.83 and 15.83 *µ*M concentration, respectively [44]. Furthermore, granaxylocarpins A and B showed weak cytotoxic effect against the P-388 murine leukemia cell lines at IC_50_ values of 9.3 and 4.9 *µ*M, respectively, but inactive against the A549 cell line (IC50 values > 10 *µ*M). In addition, granaxylocarpins C, *D*, and *E* were inactive against both the P-388 and A-549 cell lines [30]. Besides, antitumor activities of thaixylogranins A–H exhibited weak cytotoxicity against the breast MDA-MB-231 cell line [61], with the concentration of IC_50_ values of 49.4, 58.3, 53.6, 61.1, 57.9, 44.6, 40.6, and 38.5 mM, respectively, whereas thaixylogranin E showed weak cytotoxicity against the HCT-8/T cell with an IC_50_ value of 36.4 mM. Compound thaixylogranins C and D exhibited weak cytotoxicity against the melanoma A375 cell with IC_50_ values of 47.1 and 41.9 mM, respectively; and in gastric cancer AGS cell line, thaixylogranins C and D showed same cytotoxic effect with IC50 values of 41.7 and 35.0 mM, respectively [29]. Xylogranin B was isolated from *X. granatum* leaves, could inhibit T cell factor (TCF)/*β*-catenin transcriptional activity at IC_50_ 48.9 nM, and exhibited strong cytotoxicity against colon cancer cell lines. Xylogranin B drastically attenuated *β*-catenin protein; these results indicated that Wnt signal inhibitory effects [26]. All of these compounds were isolated from different parts of *X. granatum. Xylocarpus granatum* leaf extracts (ethyl acetate and its 1–7 fractions) had anticancer activity against HeLa (human cervical adenocarcinoma), T47D (breast cancer), and HT-29 cell (human colorectal adenocarcinoma cell line), with fraction 5 having the most powerful activity of 23.12 ppm IC_50_ value. However, it was concluded that, to understand the mechanism, further studies are essential [62].

#### 3.5.2. Antimalarial Activity

Mosquitoes are the key vectors for ruining parasites and pathogens including malaria, dengue, filariasis, yellow fever, chikungunya, encephalitis, and so on [63]. Malaria is a global health problem, and about 300–500 million people are infected, while almost 1 million people die annually. Natural products may be a choice for the treatment of malaria [64]. The isolated compounds from *X. granatum* plant had potential antimalarial activity [65]. The compounds gedunin and xyloccensin I, isolated from *X. granatum*, had antimalarial activity at the concentration of 50 *µ*g m/L only and showed a minimum inhibitory concentration (MIC) of 10 *µ*g m/L. This antimalarial activity was exhibited by killing the parasites in *in vitro* model of *Plasmodium falciparum* [12].

#### 3.5.3. Antiviral Activity

A virus is a particle that replicates within the living cells of an organism. Viruses can infect all types of life forms, including animals, plants, and microorganisms (like bacteria and archaea). The medicinal plant should be a good source of antiviral agents. *X. granatum* plant extract contains a variety of bioactive compounds that act against virus including sundarbanxylogranins B and granatumin L [27, 39]. Hence, sundarbanxylogranins B showed moderate effect against human immunodeficiency virus (HIV) with the concentration of 20 *µ*M; it showed a moderate inhibitory rate of 58.14 ± 3.67% and the values of IC_50_ and CC_50_ for sundarbanxylogranin B were 23.14 ± 1.29 and 78.45 ± 1.69 *µ*M, respectively [27]. Besides, *in vitro* antiviral activities of granatumin L and its derivatives against HIV-1 and influenza A virus (IAV) were evaluated. Granatumin L and their derivatives exhibit activities against the HIV-1 with an IC_50_ value of 15.98 *±* 6.87 *µ*M and a CC_50_ value greater than 100.0 *µ*M, whereas its derivative showed significant inhibitory activity against IAV with an IC_50_ value of 14.02 *±* 3.54 *µ*M and CC_50_ value greater than 100.0 *µ*M. Thus, it was inferred by the authors that alkyl groups at the C-3 position helped in exhibiting the antiviral activity against HIV [39].

#### 3.5.4. Antifeedant Activity

Some plants are used to treat several diseases and disorders. Antifeedant agents are natural substance, which stops or inhibits feeding by a pest, especially an insect [66]. Natural compounds should be the trusted source to control pests. *X. granatum* plant contains a number of isolated compounds, like secondary metabolites, and has the defense capability [67]. Several phytoconstituents and xylogranatins F, G, and R are isolated from seeds of the Chinese mangrove, *X. granatum* plant. These compounds exhibit good antifeedant activity against third instar larvae of *Mythimna separata* (Walker) at 1 mg/mL concentration [38]. Among of them, xylogranatin G was the most potent compound at 0.31 and 0.30 mg/mL concentration and 24 and 48 h; it showed 50% antifeedant activity median antifeedant concentration (AFC50), respectively [38]. Furthermore, both xyloccensins P and Q, isolated from *X. granatum* plant, showed potent antifeedant activity at 500 ppm concentration against third instar larvae of *M. separata*, whereas other compounds xyloccensins O and R–V showed weak activity [10].

#### 3.5.5. Antidiabetic Activity

Diabetes is a condition, in which the body's blood glucose is higher than the normal level [68]. Blood glucose is controlled by a vital hormone called insulin and depending on insulin the diabetes is divided into two major categories: types 1 and 2 diabetes [68, 69]. The isolated compounds from the *X. granatum* have antidiabetic activity. Xylogranin B, xyloccensin I, and xyloccensin S [70] exhibited antidiabetic activity by inhibiting *α*-amylase, *α*-glucosidase, and protein tyrosine phosphatase 1B (PTP1B), respectively [4, 52]. Xylogranin B acts with the concentration of the IC_50_ 48.9 nM or inhibited TCF/*β*-catenin transcriptional activity with IC_50_ values of 270 and 330 nM [4, 26]. Besides this other compound, xyloccensin S can control blood glucose levels with the IC_50_ value of 8.72 *µ*g/mL in PTP1B *in vitro* study [52]. In addition, xyloccensin I exhibited a hypoglycemic effect on *α*-amylase and *α*-glucosidase inhibition study at the concentrations of 0.25 and 0.16 mg/mL, respectively [4]. Hence, compounds present in the *X. granatum* have inhibitory effect on the enzymes (*α*-amylase and *α*-glucosidase) that increase the level of blood glucose in body. Inhibition of *α*-amylase and *α*-glucosidase plant extracts lead to reduction in the level of blood sugar and helps in management of diabetic condition [71–73].

#### 3.5.6. Antidepressant- and Anxiolytic-Like Activities

Anxiety and depression are generally a normal reaction to stress and there will always be situations that create stress and discomfort in humans for several reasons [74]. These disorders are currently considered the most common psychiatric illnesses affecting humans [75]. It is one of the most common psychiatric disorders. Information collected from the WHO states that depression is expected to become the second leading cause of disease-related disability by the year 2020, following heart disease [76]. Current pharmacological interventions suggest that the drugs used to manage these disorders, often have a number of side effects, including drug interactions, delayed response, and even nonresponse to the treatment [77]. Natural compounds have potential antidepressant- and anxiolytic-like activities. Recent studies exhibited that cipadesin A extracted from the fruits of the *X. granatum* plant assert potential antidepressant- and anxiolytic-like activities [2]. In the forced swimming test (FST), cipadesin A treatment significantly decreased the floating time in *in vitro* testing model. Cipadesin A treatment (15 and 50 mg/kg doses) drastically reduced the floating time [2]. Moreover, in the tail suspension test, administering 15 and 50 mg/kg doses cipadesin A significantly decreased the immobility time. Furthermore, at 5, 15, and 50 mg/kg doses significantly increased the time spent in the central zone of mice. Additionally, cipadesin A at 15 and 50 mg/kg doses significantly decreased serum corticosterone and adrenocorticotropic hormone levels [2]. The study found that after seven days, cipadesin A administered orally exhibited significant antidepressant-like effect in the tail suspension and forced swimming tests in mice [2].

#### 3.5.7. Antifilarial Activity

Filariasis is a parasitic disease caused by an infection with roundworms of the Filarioidea type [78]. These are spread by blood-feeding insects such as black flies and mosquitoes [79]. They belong to the group of diseases called helminthiases. Plants may be an effective source of antifilarial agents. Research findings proposed that photogedunin isolated from the fruits of the *X*. *granatum* plant administered by a subcutaneous route at IC50 of 0.239 and 0.213 *μ*g/mL and CC50 of 212.5 and 262.3 *μ*g/mL, respectively, at 5 × 100 mg/kg revealed excellent antifilarial efficacy, resulting in the death of 80% and 70% transplanted adult Brugia malayi in the peritoneal cavity of jirds, respectively [56].

#### 3.5.8. Antifungal Activity

Fungus infection is a major global health problem, and these life-threatening causative agents create approximately 1.5 billion deaths annually [80]. To prevent this infection, we found out some phytochemicals from natural plants. Lactone isolated from leaves of *X. granatum* plant showed 67.4% inhibition rate, and a strong fungicidal activity was proved against wheat powdery mildew with the 20 mg/mL concentration [22]. The petroleum ether and ethyl acetate extracts of *X. granatum* showed the presence of tricontanol, kaempferol, and sitosterol, which can easily penetrate the cellular barrier of powdery mildew fungus and creates pore, ultimately leading to the leakage of electrolyte causing cell death.

#### 3.5.9. Different Inhibitory Effects

The inhibitory activity was shown against PTP1B by xylogranatopyridines A and B isolated from the twigs and leaves of *X. granatum* plant. The inhibitory concentration of the chemical was an IC_50_ value of 22.9 *μ*M [52]. At the concentration of 10.0 *μ*M, krishnagranatins G, H, and I drastically inhibited the activation of nuclear factor- (NF-) *κ*B, induced by lipopolysaccharides (LPS) at the concentration of 100 ng/mL [28]. However, these compounds implied that the previously mentione NF-*κ*B inhibitory activity was not related to cell death. In conclusion, krishnagranatins G, H, and I displayed a significant inhibitory effect against the activation of NF-*κ*B signaling pathways [28]. Furthermore, xyloccensin S followed inhibitory activity against PTP1B at the amount of IC_50_ value of 8.72 *μ*g/mL [36].

#### 3.5.10. Antioxidant Activity

The antioxidant constituents from ethanol bark extract of a medicinally important mangrove plant *X. granatum* [4]. Limonoid derivative xyloccensin I showed antioxidant activity in 2,2-diphenyl-1-picrylhydrazyl (DPPH), 2,2′-azino-bis(3-ethylbenzothiazoline-6-sulfonic acid) (ABTS), superoxide, and hydrogen peroxide scavenging studies at IC50 values of 0.041, 0.039, 0.096 and 0.235 mg/mL, respectively [4]. In a recent study by Das and coworkers [81], demonstrated that bark ethanolic extract reflected highest ABTS scavenging activity with IC_50_ value of 41.50 𝜇g/mL, whereas butylated hydroxyl toluene (standard antioxidant) demonstrated antioxidant activity of 76.34 𝜇g/mL. *In vivo* antioxidant analysis showed that enzymatic antioxidants such as superoxide dismutase, catalase, and glutathione reductase in liver and brain tissue of diabetic mice increased when supplemented with 200 mg/kg of *X. granatum.* Hence, it was concluded that increase in the antioxidant defense system helped the diabetic mice in overcoming the oxidative stress.

#### 3.5.11. Antibacterial Effect

Stem bark extracts (ethanol extract, pet-ether fraction, CCl4 fraction, and CHCl3 fraction) from *Xylocarpus granatum* depicted antimicrobial activity against *Staphylococcus epidermis* (20–25 mm), *Staphylococcus aureus* (20–25 mm)*, Shigella boydii* (20–25 mm)*, Proteus spp.* (20–25 mm)*, Escherichia coli* (20–25 mm)*, and Streptococcus pyogenes* (20–25 mm) in terms of disc inhibition zone (diameter in mm) at concentration of 400 𝜇g/disc. However, the exact mechanism is not known [82].

#### 3.5.12. Antidiarrheal Effect

*Xylocarpus granatum* bark extracts (methanol extracts) when supplemented in mice induced with diarrhea (induced using castor oil and magnesium sulphate) revealed that, at oral dosage of 250 and 500 mg/kg, it exhibited antidiarrheal properties by reducing the wet faeces discharge. Castor oil is known to cause diarrhea due to its hypersecretory activity caused by active component ricinoleic acid, and the antidiarrheal activity of the *Xylocarpus granatum* bark extracts could be due to its antisecretory effect [83].

These studies, highlighted in the present review on the different pharmacological activities exhibited by parts of *Xylocarpus granatum*, its extracts, and bioactive compounds, indicate the health promoting effects of *Xylocarpus granatum*, which thus justifies their application as indigenous medicine in different traditional medicinal system used across the globe. It also paves way for further research to translate these natural plant-based bioactive compounds as advanced pharmaceutical drugs for treating various disorders, thus allowing researchers to explore the best of both scientific as well as traditional knowledge systems.

## 4. Toxicity

Limited research is available on the toxicity of *X. granatum* and its extracts. However, a study depicted that oral dosage of ethanolic bark extract of *X. granatum* at 1000 mg/kg body weight per day when given to healthy Balb/c mice showed no signs of toxic effects or death up to four days [81]. Another study indicated that ethyl acetate extract of *X. granatum* leaves had no toxicity when tested using brine shrimp lethality test (BSLT) even above 1500 ppm concentration [62]. In conclusion, though few studies indicate no toxicity, detailed experiments are necessary to further establish the toxicity or upper tolerable limits.

## 5. Conclusion and Future Prospects

*X. granatum* may be one of the hopeful medicinal herbs for the treatment of various diseases in humans. Traditionally, this plant was widely used in treating several diseases, because of its chemical constituents. Several studies have shown that *X. granatum* has anticancer, antiviral, antidepressant, antifeedant, and antimalarial activities ascribed to its chemical constituents such as limonoids, phragmalin, limonoid-based alkaloids, mexicanolides, protolimonoids, flavonol-like compounds, and alkaloids, among others. These chemical compounds are essential to treat many diseases and should be established as standard drugs for several known physiological disorders and diseases in medicinal chemistry and pharmacology. Still there is a lack of clinical trials on utilization of *X. granatum* and its bioactive compounds or extracts, and fewer studies are conducted on exploiting the development of plant-based drugs using *X. granatum*. Thus, more research is necessary to understand its chemical compounds and utilization as novel drugs in human studies and investigate the mechanism of action in treating various ailments. Also, the toxicological aspects of this medicinal mangrove plant need to be investigated thoroughly before developing any novel drug as limited studies are available.

## Figures and Tables

**Figure 1:** Different parts of Xylocarpus granatum J Koenig. (a) Leaves, (b) flowers, (c) unripe fruit, (d) ripe fruit, (e) stem and bark, and (f) roots.

**Figure 2:** Chemical constituents of *Xylocarpus granatum* J. Koenig.

**Table 1:** Phytochemistry of *Xylocarpus granatum* J. Koenig.

Parts	Compounds	References
Seeds	Sundarbanxylogranins A–E; krishnagranatins A–I; thaixylogranins A–H; granaxylocarpins A–E; xylocarpanoids A and B; xylomexicanins A–D, I, and J; xyloccensin I, K, L, O–S, V, W, and Y; hainangranatumins A–J; xylogranatins F–R; thaigranatins A–E; xylocartin C; andhraxylocarpins A–E; protoxylogranatin A-B; protoxylocarpins F–H	[10, 12, 25, 27–43]
Stem bark	Xyloccensin M and N; xyloccensins Q–U; xyloccensin L; xyloccensin I, J; xyloccensins O and P	[10, 44–47]
Fruits	Gedunin; andirobin; mexicanolide; phragmalin; cipadesin A; xylocarpins A–I; photogedunin, xylocarpin L, xyloccensin I, Y, X1, and X2; xylogranatin E; xylogranatinin	[2, 8, 16, 35, 40, 48–51]
Leaf and twigs	Lactone; xyloccensins O–S and V; xylogranin B; xylogranatopyridines A and B; xylogranatumines A–G; xylogranatin E	[22, 26, 36, 50, 52, 53]
Root bark	N-Methylflindersine	[54]

**Table 2:** Pharmacological activities.

Activity	Isolated compounds	Cell lines/test system	IC_50_ values	References
Anticancer activity	Gedunin	Colon cancer cell lines	16.83 *µ*M	[16]
	Xylogranatumines A–G	A549 (human lung adenocarcinoma) tumor cell lines	10 *µ*M per specimen	[53]
	Protoxylocarpins F–H	Five human tumor cell lines		[25]
	Xylomexicanin A	Human breast carcinoma cells (KT)	7.43 *µ*M	[32]
	Granaxylocarpins A-E	Cytotoxicity against the P-388 and A-549 tumor cell lines	9.3 and 4.9 *µ*M	[30]
	Xylomexicanins F	Six human tumor cell lines A549 and RERF	18.83 and 15.83 *µ*M	[44]
	Thaixylogranis A–H	MDA-MB-231 cell line	49.4 mM	[29]
	Xylogranin B		48.9 nM	[26]

Antimalarial activity	Gedunin and xyloccensin I	*In vitro* model of *Plasmodium falciparum*	50 µg m/L, and (MIC) 10 *µ*g m/L.	[12]

Antiviral activity	Sundarbanxylogranis B	Human immunodeficiency virus (HIV)	78.45 ± 1.69 *µ*M.	[27]
	Granatumin L and their moderate derivatives	HIV-1 and influenza A virus (IAV)	HIV-1 with an 15.98 ± 6.87 *µ*M; IAV with a 14.02 ± 3.54 *µ*M	[39]

Antifeedant activity	Xylogranatins G	The third instar larvae of *Mythimna separata* (walker)	1 mg m/L	[38]
	Xyloccensins P and Q		500 ppm	[10]

Antidiabetic activity	Xylogranin B		IC_50_ 48.9 nM or inhibited TCF/*β*-catenin transcriptional activity with IC50 values of 270 and 330 nM	[26]
	Xyloccensin I	*α*-amylase and *α*-glucosidase inhibition study	0.25 and 0.16 mg/mL	[4]
	Xyloccensin S	Protein tyrosine phosphatase 1B	8.72 *µ*g/mL	[52]

Antidepressant- and anxiolytic-like activities	Cipadesin A	Mice model	5, 15, and 50 mg/kg	[2]

Antifilarial activity	Gedunin and photogedunn	Human lymphatic filarial parasite	100 mg/kg	[56]

Fungicidal activity	Lactone	Wheat powdery mildew	20 mg/mL	[22]

Possess different inhibitory effect	Xylogranatopyridins A and B	Protein tyrosinephosphatase 1B (PTP1B)	22.9 *µ*M	[52]
	Krishnagranatins *G*, H, and I	Inhibit NF-*κ*B pathway	100 ng/mL	[28]
	Xyloccensin S	Protein tyrosine phosphatase 1B	8.72 *µ*g/mL	[36]

Antioxidant activity	Xyloccensin I	DPPH, ABTS, superoxide and hydrogen peroxide scavenging	0.041, 0.039, 0.096, and 0.235 mg/mL	[4]
